The article "Therapeutic Effect and Prognosis of PiCCO in the Treatment of Myocardial Injury Complicated with Septic Shock" was published in 2022. Journal: Comput Math Methods Med.

# Therapeutic Effect and Prognosis of PiCCO in the Treatment of Myocardial Injury Complicated with Septic Shock

**DOI:** 10.1155/2022/2910849

**Published:** 2022-06-06

**Authors:** Xuan Lu, Huaixiang Zhai, Yue Dong, Fei Su, Yongpeng Xie, Yanli Wang, Lili Wang, Jiguang Li, Ping Xu

**Affiliations:** ^1^Emergency Intensive Care Unit, Lianyungang Clinical College of Nanjing Medical University, The First People's Hospital of Lianyungang, Jiangsu, China; ^2^Intensive Care Unit, The First People's Hospital of Lianyungang, Jiangsu, China; ^3^Emergency Intensive Care Unit, The First People's Hospital of Lianyungang, Jiangsu, China; ^4^Department of Emergency and Critical Medicine, The First People's Hospital of Lianyungang, Jiangsu, China

## Abstract

**Objective:**

To explore the effect of pulse-induced contour cardiac output (PiCCO) monitoring on the survival and prognosis of patients with myocardial injury and septic shock.

**Methods:**

A total of 400 patients with MI and septic shock who were treated in our hospital from May 2018 to June 2021 were included in the study. They were randomly grouped into the PiCCO group (*n* = 200) and the control group (*n* = 200) according to whether PiCCO was used for monitoring during the treatment period. The clinical baseline characteristics of all the patients were recorded. For comparison, we recorded hemodynamic parameters including mean arterial pressure (MAP), central venous pressure (CVP), heart rate (HR), troponin I (TnI), brain natriuretic peptide (BNP), oxygen metabolism parameters including systemic central venous oxygen saturation (ScvO_2_), and lactate before and 6 h after intervention. In addition, white blood cell count (WBC) and C-reactive protein (CPR) levels before and 6 h, 24 h, 48 h, and 72 h after intervention were measured in both groups. Finally, the survival and prognostic parameters were compared between the two groups.

**Results:**

At 6 h after monitoring intervention, the hemodynamic parameters of the patients in the PiCCO group were significantly increased. Additionally, compared with the control group, the ScvO_2_ level was higher while the lactate level was lower in the PiCCO group. An intergroup comparison on inflammation also showed that WBC and CPR levels recovered better in the PiCCO group than in the control group. Moreover, patients with PiCCO monitoring showed better performance in outcome measures such as mortality, duration of invasive mechanical ventilation, length of hospital stay, duration of ventilator use, acute physiology and chronic health scores, and postoperative complications.

**Conclusion:**

With the monitoring and guidance of the PiCCO technique, the nursing outcomes, survival rate, and prognosis of patients with myocardial injury and septic shock can be improved.

The article "Therapeutic Effect and Prognosis of PiCCO in the Treatment of Myocardial Injury Complicated with Septic Shock" was published in 2022. Journal: Comput Math Methods Med.

## 1. Introduction

Myocardial injury, according to the causes, can be clinically divided into ischemic or nonischemic [1]. The prevalence of ischemic myocardial injury has been increasing, and consequently, heart diseases caused by myocardial ischemia, such as myocardial infarction or ischemic heart failure, are the leading causes of mortality in the developed countries [2]. Similarly, an increasing prevalence of nonischemic myocardial injury has been reported. Antithrombotic therapy and percutaneous coronary intervention are the standard treatment approaches for nonischemic myocardial injury [3, 4]. However, patients may develop postoperative infection and even septic shock as a complication of percutaneous coronary intervention. Septic shock can cause multiple organs and system injuries (such as heart, respiration, kidney, liver, blood, and central nervous systems injuries) and easily lead to myocardial infarction and cardiac depression [5].

Myocardial dysfunction includes low cardiac output or systolic/diastolic ventricular dysfunction after sudden cardiac arrest, and nearly two-thirds of patients resuscitated after sudden cardiac arrest are reported to have impaired left ventricular systolic function [6]. Therefore, in such cases, hemodynamic monitoring at all times is critical. Pulse-induced contour cardiac output (PiCCO) technology is an efficient and advanced system for monitoring the hemodynamic status of patients with septic shock in the intensive care unit (ICU). The continuous hemodynamic monitoring with PiCCO was achieved via the insertion of large arterial (femoral, brachial, or axillary) catheters and central venous catheters [7]. This technique provides continuous monitoring of parameters such as cardiac output, intrathoracic blood volume index (ITBVI), end-diastolic volume, extravascular lung water index (EVLWI), and left systolic index [7]. Previous findings have shown that compared with central venous pressure, the end-diastolic volume and ITBVI provided by PiCCO more accurately reflect cardiac preload and can better predict the patient's response to fluid resuscitation therapy [8]. However, there are only a few relevant studies on the effects of PiCCO monitoring on the survival and prognosis of patients with myocardial injury and septic shock. Therefore, this study explored the usefulness of PiCCO in accelerating the rehabilitation of patients with myocardial injury and septic shock and therefore improving their prognosis and survival rate.

## 2. Materials and Methods

### 2.1. Study Subjects

A total of 400 patients with myocardial injury septic shock complications who received treatment in our hospital from May 2018 to June 2021 were analyzed retrospectively. They were randomly divided into the PiCCO monitoring group (PiCCO, *n* = 200) and a control group, without PiCCO monitoring (control; *n* = 200). The inclusion criteria were as follows: (1) patients with myocardial injury and septic shock and over 18 years old, (2) patients who tolerated PiCCO monitoring, and (3) patients who gave informed consent and volunteered to participate in this study. The exclusion criteria were as follows: (1) patients with malignant tumors, (2) patients with mental illnesses, (3) patients with severe liver and kidney dysfunction, and (4) patients with other severe cardiovascular and cerebrovascular diseases. The clinical baseline characteristics of all the patients were recorded, including age, sex, height, weight, number of primary infections, and other information. The study conformed to medical ethical standards and was approved by the Medical Ethics Committee of the First People's Hospital of Lianyungang (No. LCYJ20180427002).

The article "Therapeutic Effect and Prognosis of PiCCO in the Treatment of Myocardial Injury Complicated with Septic Shock" was published in 2022. Journal: Comput Math Methods Med.

### 2.2. Interventions

PiCCO monitoring was done in the PiCCO group. Fluid resuscitation was guided by the ITBVI and cardiac index (CI) to achieve an ITBVI of 850-1000 mL/m^2^ and CI ≥ 2.5 L/min·m^2^; dobutamine or milrinone was used to regulate cardiac function if ITBVI was >1000 mL/m^2^, but CI was still <2.5 L/min·m^2^ or the left ventricular maximum systolic force index (dPmax) was reduced. The dose of norepinephrine was adjusted according to the systemic vascular resistance index (SVRI) to steadily maintain mean arterial pressure (MAP) at ≥65 mmHg. Fluid selection and diuretic use were guided by the EVLWI; if central venous oxygen saturation (ScvO_2_) < 70% and hematocrit (HCT)<30%, red blood cells were transfused to make HCT ≥ 30%.

Conventional treatment was administered in the control group. Fluid resuscitation was guided by early goal-directed therapy (EGDT): volume expansion fluid was given to hypotensive patients within 30 min until central venous pressure (CVP) was ≥2 mmHg; if MAP was <70 mmHg, norepinephrine was used to maintain a MAP of ≥70 mmHg; if HCT was <30% and ScvO_2_ < 70%, red blood cells were transfused to make HCT ≥ 30%. The treatment goals were achieved if the following were attained: CVP 8-12 mmHg, MAP 70-90 mmHg, ScvO_2_ ≥ 70%, and urine volume ≥ 0.5 mL/(kg·h). The operational process is shown in Figure 1.

### 2.3. Hemodynamic Parameters

The following hemodynamic parameters were observed before intervention and 6 h after the intervention, including MAP, CVP, heart rate (HR), serum myocardial necrosis marker (TnI), and serum B-type natriuretic peptide (BNP).

The article "Therapeutic Effect and Prognosis of PiCCO in the Treatment of Myocardial Injury Complicated with Septic Shock" was published in 2022. Journal: Comput Math Methods Med.

### 2.4. Oxygen Metabolism Indexes

The oxygen metabolism indexes, including ScvO_2_ and lactate levels, were recorded before intervention and 6 h after intervention.

### 2.5. Inflammation-Related Parameters

White blood cell count (WBC) and C-reactive protein (CRP) levels were measured before and 6 h, 24 h, 48 h, and 72 h after intervention in both groups.

### 2.6. Survival Outcome Indicators

Survival and prognostic indicators were recorded after the intervention, including the number of deaths, duration of invasive mechanical ventilation, ICU stay, length of hospital stay, duration of ventilator use, acute physiology and chronic health scores, and postoperative complications.

### 2.7. Statistical Analysis

Data were statistically analyzed using SPSS 26.0 software. Measurement data conformed to normal distribution were expressed as the mean ± standard deviation (SD). An independent sample *t*-test was used to compare measurement data of the two groups and a chi-square test for comparing enumeration data between the groups. *P* < 0.05 was considered statistically significant.

## 3. Results

### 3.1. General Patients' Characteristics

A total of 200 were analyzed, and the majority were males, but there was no significant difference in the number of males and females between the groups. There were no significant differences in mean age, height, and weight between the two groups. In addition, there were no significant differences in serum parameters TnI, BNP, ScvO_2_, lactate, WBC, and CRP levels between the two groups (Table 1). Therefore, the two groups were comparable.

### 3.2. Comparison of Hemodynamic Parameters between the Two Groups

The hemodynamic parameters were compared between the two groups before and 6 hours after the intervention. The results showed no significant differences in hemodynamic parameters between the two groups before the intervention. However, at 6 h after the intervention, the hemodynamic parameters of both groups were increased compared with those before the intervention. In addition, patients in the PiCCO group had a significantly higher MAP (85.10 ± 4.97), CVP (9.87 ± 1.06), HR (96.43 ± 5.41), TnI (29.20 ± 1.97), and BNP (957.72 ± 55.26) than those in the control group at 6 h after intervention (Figures 2(a)–2(e)).

### 3.3. Comparison of Oxygen Metabolism Parameters between the Two Groups

The oxygen metabolism parameters were further compared between the two groups. As shown in Figures 3(a) and 3(b), there were no significant differences in ScvO_2_ and lactate before intervention between the two groups. However, 6 hours after intervention, ScvO_2_ levels were significantly higher in the PiCCO group (85.94 ± 5.52) than in the control group (75.42 ± 4.93), and the lactate levels were lower in the PiCCO group (2.10 ± 0.54) compared with the control group (2.72 ± 0.51).

The article "Therapeutic Effect and Prognosis of PiCCO in the Treatment of Myocardial Injury Complicated with Septic Shock" was published in 2022. Journal: Comput Math Methods Med.

### 3.4. Comparison of Inflammatory Factor Levels at Different Times between the Two Groups

WBC and CPR concentrations in the serum of patients in both groups were measured. The results showed that the concentrations of the two were gradually upregulated in both groups after intervention. Further, a postintervention intergroup comparison revealed that WBC and CPR concentrations were significantly higher in the PiCCO group than in the control group at 6 h, 24 h, 48 h, and 72 h after intervention (Figures 4(a) and 4(b)).

### 3.5. Comparison of Survival Outcome Indicators between the Two Groups

The survival and prognosis of patients in the two groups were further analyzed. The results showed a significantly lower mortality rate in the PiCCO group (13.5%) than in the control group (24%). In addition, compared with the control group, PiCCO monitoring was associated with a shorter duration of invasive mechanical ventilation, ICU stay, hospital stay, and ventilator time. Also, the acute physiology and chronic health scores and the incidence rate of postoperative complications in the PiCCO group were significantly lower than those in the control group. These results indicated that the posttreatment use of PiCCO monitoring promoted rehabilitation and improved the prognosis of patients with myocardial injury and septic shock (Table 2).

Values are *n* (%) or mean ± SD.

## 4. Discussion

Myocardial injury with septic shock complication is an important cause of death in critically ill patients in the ICU [9]. Absolute or relative insufficiency of circulating blood volume can present patients with myocardial injury with 9+ complications, resulting in hemodynamic instability [10]. It has been reported that the optimal treatment of myocardial dysfunction with septic complications includes proper and timely management of infection, optimization of hemodynamic parameters, and subsequent effective fluid resuscitation [11]. Therefore, advanced hemodynamic monitoring remains a cornerstone in the management of myocardial injuries with septic complications. EGDT proposed by Rivers et al. focuses on the rapid increase of cardiac output and oxygen flow, immediate restoration of circulating blood volume, and reduction in the time of tissue and organ hypoperfusion [12]. However, hemodynamic management in strict accordance with the EGDT protocol in septic shock patients detected early, receiving intravenous antibiotics and adequate fluid resuscitation, may not improve prognosis [13]. It is, therefore, crucial to find other efficient and accurate protocols for monitoring hemodynamics. PiCCO monitoring, an alternative to pulmonary artery catheter monitoring of cardiac output, can integrate a large amount of static and dynamic hemodynamic data through a combination of transcardiopulmonary thermoregulation and pulse contour analysis [14]. PiCCO can fully reflect the changes in hemodynamic parameters, as well as the systolic and diastolic function, so it is beneficial in fluid resuscitation, fluid management, and clinical application [15]. Therefore, in this study, we compared the clinical nursing effects of two different interventions in patients with myocardial injury and septic shock. Our results showed that at 6 h after the intervention, patients in the PiCCO group had significantly higher levels of hemodynamic parameters (MAP, CVP, HR, TnI, and BNP) than those in the control group.

The article "Therapeutic Effect and Prognosis of PiCCO in the Treatment of Myocardial Injury Complicated with Septic Shock" was published in 2022. Journal: Comput Math Methods Med.

Early sepsis and septic shock are characterized by abnormal circulation that is often associated with hypovolemia and vasodilation and consequently a potential imbalance between oxygen supply and demand in various organs [16]. Both TNF-*α* and IL-1*β* are major players in the hierarchy of proinflammatory mediator cascades [17], while nitric oxide (NO) and oxygen free radicals are secondary effectors of cardiac depression in systemic inflammatory response syndromes [11]. Sepsis has been reported to affect the expression of inducible nitric oxide synthase (iNOS) in the myocardium leading to high levels of NO and consequently myocardial dysfunction and increased total sarcoplasmic reticulum Ca^2+^ load and myofilament sensitivity to Ca^2+^ [18]. These inflammatory factors have a direct inhibitory effect on cardiomyocyte contractility, resulting in systolic and diastolic dysfunction in septic cardiomyopathy. Moreover, the enhanced intensity of the inflammatory response in septic shock leads to a higher mortality rate [19]. In animal models, treatment with corticosteroids and other drugs has been shown to reduce myocardial dysfunction after cardiopulmonary bypass [20]. The results of this study showed that ScvO_2_ was significantly increased in patients after PiCCO intervention while lactate levels were significantly decreased. Additionally, the recovery of inflammatory factor levels in the PiCCO group was better than in the control group. After follow-up, we also found that patients monitored with PiCCO had a significantly better prognosis, with a shorter duration of invasive mechanical ventilation, ICU stay, hospital stay, ventilator time, and lower incidence of postoperative complications. Together, these results showed that PiCCO can provide highly accurate information for clinical nursing and is a valuable approach that should be widely popularized and utilized.

The article "Therapeutic Effect and Prognosis of PiCCO in the Treatment of Myocardial Injury Complicated with Septic Shock" was published in 2022. Journal: Comput Math Methods Med.

Our study had several limitations. First, it was a single-center study and may not be an accurate representation of myocardial injury with septic shock complication cohort in other regions. Second, it was retrospective in nature. Third, while medications are important factors influencing prognosis and survival outcomes, the effects of medication-related factors were not analyzed. Further research study including more potential influencing factors and different patient populations is required.

## 5. Conclusion

With the monitoring and guidance of PiCCO monitoring technology, the nursing outcomes, prognosis, and survival rate of patients with myocardial injury and septic shock can be improved. However, this study is a single-center clinical trial and has limitations. Further research is required to provide a more comprehensive data basis for the clinical application of PiCCO.

## Figures and Tables

**Figure 1:** The flow chart of PiCCO monitoring.

**Figure 2:** Comparison of hemodynamic parameters between the PiCCO and control groups before and after intervention. Changes in MAP (a), CVP (b), HR (c), TnI (d), and BNP (e) levels before and 6 h after intervention in both groups. ^∗^*P* < 0.05 vs. control; ^#^*P* < 0.05 vs. 0 h. MAP: mean arterial pressure; CVP: central venous pressure; HR: heart rate; TnI: troponin I; BNP: serum B-type natriuretic peptide.

**Figure 3:** Comparison of oxygen metabolism parameters before intervention and at 6 h after intervention between the two groups. (a) ScvO_2_ levels before and 6 hours after intervention in both groups; (b) lactate levels before and 6 hours after intervention in both groups. ^∗^*P* < 0.05 vs. control; ^#^*P* < 0.05 vs. 0 h. ScvO_2_: systemic central venous oxygen saturation.

**Figure 4:** Comparison of inflammatory factor levels at different times between the two groups. Comparison of WBC (a) and CPR (b) concentrations before intervention and 6 h, 24 h, 48 h, and 72 h after intervention between the two groups. ^∗∗∗^*P* < 0.001 vs. control. WBC: white blood cell count; CPR: C-reactive protein.

**Table 1:** Baseline data of the patients.

	PiCCO group (*n* = 200)	Control group (*n* = 200)	*χ* ^2^/*t*	*P*
Sex (M/F, *n* (%))	133/67	122/78	1.309	0.253
Age (year)	59.42 ± 5.08	60.16 ± 5.03	-1.454	0.147
Height (cm)	170.71 ± 8.59	169.70 ± 9.05	1.145	0.253
Weight (kg)	76.16 ± 18.76	75.30 ± 15.58	0.499	0.618
Number of primary cases (n)	67/133	84/116	3.075	0.080
Mean arterial pressure (MAP, mmHg)	65.98 ± 4.28	66.21 ± 4.59	-0.529	0.597
Central venous pressure (CVP, kPa)	6.59 ± 0.78	6.72 ± 0.91	-1.496	0.135
Heart rate (HR, bpm)	76.70 ± 5.25	76.41 ± 5.13	0.549	0.583
Troponin I (TnI, ng/L)	25.00 ± 1.67	25.01 ± 1.53	-0.081	0.936
Serum B-type natriuretic peptide (BNP, pg/mL)	853.16 ± 54.72	849.54 ± 51.07	0.684	0.494
Central venous oxygen saturation pressure (ScvO_2_, %)	64.54 ± 2.35	64.37 ± 2.36	0.717	0.473
Lactate level (mmol/kg)	4.06 ± 0.55	4.10 ± 0.55	-0.608	0.543
White blood cell (WBC, 10^9^/mL)	6.02 ± 0.11	6.03 ± 0.11	-0.611	0.542
C-reactive protein (CRP, mg/L)	2.50 ± 0.21	2.49 ± 0.21	0.652	0.515

The article "Therapeutic Effect and Prognosis of PiCCO in the Treatment of Myocardial Injury Complicated with Septic Shock" was published in 2022. Journal: Comput Math Methods Med.

**Table 2:** Comparison of survival outcome indicators between the two groups.

	PiCCO group (*n* = 200)	Control group (*n* = 200)	*χ* ^2^/*t*	*P*
Mortality rate (%)	27 (13.5%)	48 (24%)	7.237	0.007
Duration of invasive mechanical (d)	17.20 ± 1.35	23.69 ± 3.20	-26.459	≤0.001
ICU stay (d)	25.97 ± 1.33	32.38 ± 3.77	-22.636	≤0.001
Hospital stay (d)	47.34 ± 4.85	53.44 ± 7.30	-9.839	≤0.001
Ventilator duration (d)	22.42 ± 1.71	28.89 ± 3.15	-25.566	≤0.001
Acute physiology and chronic health scores	21.00 ± 2.06	27.36 ± 3.14	-23.970	≤0.001
Cases with postoperative complications (*n*)	30 (15%)	70 (35%)	23.214	≤0.001

## Data Availability

The data used to support the findings of this study are available from the corresponding author upon request.
